# Pinosylvin Extract Retinari™ Sustains Electrophysiological Function, Prevents Thinning of Retina, and Enhances Cellular Response to Oxidative Stress in NFE2L2 Knockout Mice

This article has been retracted.

**DOI:** 10.1155/2021/8028427

**Published:** 2021-12-07

**Authors:** Toni Tamminen, Ali Koskela, Elisa Toropainen, Iswariyaraja Sridevi Gurubaran, Mateusz Winiarczyk, Mikko Liukkonen, Jussi J. Paterno, Petri Lackman, Amir Sadeghi, Johanna Viiri, Juha M. T. Hyttinen, Ari Koskelainen, Kai Kaarniranta

**Affiliations:** ^1^Department of Ophthalmology, Institute of Clinical Medicine, University of Eastern Finland, P.O. Box 1627, FI-70211 Kuopio, Finland; ^2^School of Pharmacy, University of Eastern Finland, P.O. Box 1627, FI-70211 Kuopio, Finland; ^3^Department of Vitreoretinal Surgery, Medical University of Lublin, Poland; ^4^Department of Ophthalmology, Kuopio University Hospital, P.O. Box 100, FI-70029 KYS Kuopio, Finland; ^5^Eevia Health Oy, FI-60100 Seinäjoki, Finland; ^6^Department of Neuroscience and Biomedical Engineering, Aalto University, FI-00067 Aalto, Finland

## Abstract

Chronic oxidative stress eventually leads to protein aggregation in combination with impaired autophagy, which has been observed in age-related macular degeneration. We have previously shown an effective age-related macular degeneration disease model in mice with nuclear factor-erythroid 2-related factor-2 (NFE2L2) knockout. We have also shown pinosylvin, a polyphenol abundant in bark waste, to increase human retinal pigment epithelium cell viability *in vitro*. In this work, the effects of commercial natural pinosylvin extract, Retinari™, were studied on the electroretinogram, optical coherence tomogram, autophagic activity, antioxidant capacity, and inflammation markers. Wild-type and NFE2L2 knockout mice were raised until the age of 14.8 ± 3.8 months. They were fed with either regular or Retinari™ chow (141 ± 17.0 mg/kg/day of pinosylvin) for 10 weeks before the assays. Retinari™ treatment preserved significant retinal function with significantly preserved a- and b-wave amplitudes in the electroretinogram responses. Additionally, the treatment prevented thinning of the retina in the NFE2L2 knockout mice. The NFE2L2 knockout mice showed reduced ubiquitin-tagged protein accumulation in addition to local upregulation of complement factor H and antioxidant enzymes superoxide dismutase 1 and catalase. Therefore, the treatment in the NFE2L2 KO disease model led to reduced chronic oxidative stress and sustained retinal function and morphology. Our results demonstrate that pinosylvin supplementation could potentially lower the risk of age-related macular degeneration onset and slow down its progression.

## 1. Introduction

Age-related macular degeneration (AMD) is the most common cause of blindness in the elderly in the western world. The disease is classically divided into dry (nonexudative) and wet (exudative) AMD forms. The dry form of the disease is more prevalent, accounting for up to 90% of all cases. Currently, there is no effective treatment against dry AMD, while wet AMD can be managed with intravitreal injections of antivascular endothelial growth factor (anti-VEGF) [1, 2]. The pathogenesis of AMD is multifactorial. It involves the progressive degeneration of the retinal pigment epithelium (RPE) and photoreceptors of the macular region of the eye. Chronic oxidative stress and inflammation can be considered the main molecular mechanisms involved in pathogenesis [3–5]. Furthermore, oxidative damage limiting system dysfunction and inflammation-related accumulation of lipofuscin and drusen deposits in the retina are inherently part of the pathogenesis [6, 7].

Recently, we reported that the nuclear factor-erythroid 2-related factor-2 (NFE2L2) and peroxisome proliferator-activated receptor gamma coactivator 1-alpha (PGC1-*α*) double knockout (KO) mice develop a dry AMD resembling phenotype that coincides with visual loss [8]. The NFE2L2 deficiency was responsible for the majority of molecular changes observed in the RPE cells, including oxidative stress. In its inactive state, the NFE2L2 transcription factor is bound to kelch-like ECH-associated protein 1 (Keap1) in the cytoplasm. In response to oxidative stress, NFE2L2 is released from the complex and translocated to the nucleus where it binds to the antioxidant response element (ARE) which triggers the expression of various cytoprotective genes [9–14]. However, despite the clear effects of NFEL2 deficiency on oxidative stress and disease-like phenotype, NFE2L2 signalling is not the only pathway controlling oxidative stress [15, 16]. For example, many protective antioxidative enzymes are regulated by several other factors, including activator protein 1 (AP-1) and forkhead box transcription factors of the class O (FoxO) [17].

The spontaneous decline of the NFE2L2-ARE pathway and increased oxidative stress during ageing calls for functional damage limiting pathways, including autophagy and inflammatory response [18–21]. Autophagy is a dynamic process where ubiquitin-conjugated proteins destined to degradative pathways aggregate and are sequestered to autophagosomes with the interaction between cargo receptor p62/SQSTM1 (p62) and autophagosome marker microtubule-associated protein 1A/1B-light chain 3 (LC3) [22]. Ubiquitinated proteins, cargo, and autophagosome markers are degraded later in autolysosomes formed after the fusion of autophagosome and lysosome. In the immune system, the complement system has been implicated as one factor in the pathogenesis of AMD, as reviewed recently by Armento et al. [23]. Specifically, the alternative pathway of the complement system, which is regulated by complement factor H (CFH), has been connected in part to the pathogenesis of AMD [23]. A common genetic variant, Y402H polymorphism, in the *CFH* gene is a risk factor for the development of AMD due to the role of CFH in regulating the alternative pathway [24, 25]. The complement system disbalance caused by the Y402H variant can be observed as increased chronic inflammation and accumulation of the inflammation marker C-reactive protein (CRP) in the drusen [24, 26].

Pinosylvin (3,5-dihydroxy-*trans*-stilbene) is a lipophilic polyphenolic stilbene found in Scots pine (*P. sylvesteris*). It is thought to be an analogue of resveratrol (3,4′,5-trihydroxy-*trans*-stilbene) which is the most studied polyphenolic compound. While resveratrol has been shown to combat the detrimental effects of oxidative stress and induce autophagy in human cell cultures [27–30], it has poor bioavailability. Although resveratrol is absorbed remarkably well, it is very quickly metabolized and thus has negligible systemic bioavailability [31]. Additionally, the low concentration of resveratrol in natural substances requires it to be produced in a laboratory setting which is not cost-effective. These factors have prompted the search for a cost-effective analogue of resveratrol with better bioavailability. A mere one additional hydroxyl group is present in resveratrol in comparison to pinosylvin. This difference makes pinosylvin more lipophilic with a partition coefficient log*P* of 3.5 [32], compared to resveratrol (log*P* 3.1) [33]. This would suggest that pinosylvin permeates the cell membrane better. However, the majority of orally administered stilbene compounds become metabolized before reaching the circulatory system [34]. Interestingly, one of the main metabolites of pinosylvin seems to be resveratrol [35, 36]. This opens an opportunity for pinosylvin to act as a precursor for resveratrol when administered orally.

Pinosylvin has strong protective effects in response to oxidative stress in cell cultures and animal models [37, 38]. While NFE2L2 signalling has been identified as the main target of pinosylvin in oxidative stress protection, resveratrol may enhance antioxidant defence via several other pathways including AP-1 and SIRT1 (sirtuin 1)/FoxO signalling [38–40]. Since NFE2L2 KO mice lack the *NFE2L2* gene response and exhibit AMD-like changes including oxidative stress, changes in autophagic activity, and accumulation of ubiquitin-tagged proteins in the retina [8, 41], we were curious to analyse the effects of pinosylvin in this animal model as well as wild-type (WT) animals with intact NFE2L2 signalling. We studied the electrophysiology of the visual system with ERG, morphological changes in optical coherent tomography (OCT), and antioxidant defence system functionality as well as markers of inflammation, lipid peroxidation, and autophagic protein clearance.

## 2. Materials and Methods

### 2.1. Animals

All animal protocols were approved by the Project Authorisation Board of Finland (ESAVI/8621/04.10.07/2017 on 13.12.2017) and conducted in compliance with the European Community Council Directives 2010/63/EU and ARVO statement for the Use of Animals in Ophthalmic and Vision Research. 3R principles were applied. Two types of mice were raised in the Lab Animal Centre of the University of Eastern Finland: WT and NFE2L2 KO (*NFE2L2^−/−^*), both of which were derived from C57BL/6J inbred strain. The breeding scheme involved interbreeding heterozygote *NFE2L2^+/-^* to produce WT (*NFE2L2^+/+^*), heterozygote (*NFE2L2^+/-^*), or homozygote (*NFE2L2^−/−^*) mice for the study. The heterozygote strain is regularly backcrossed with WTs from a larger population to maintain as healthy a strain as possible. The retinal degeneration 8 (rd8) mutation is absent in these subpopulations. The genotyping of these strains has been presented earlier [8]. The mice were housed in 12 : 12-hour light-dark conditions and given food and water *ad libitum*.

The mice were raised until the age of 14.8 ± 3.8 months with some selection involved to produce as homogenous a population as possible in terms of their age. 10 WT and 10 NFE2L2 KO mice were initially grown for the Retinari™ treatment trial, with each type having half assigned to the Retinari™ treatment group and the other half to the control group. The treatment was carried out with a commercial substance named Retinari™. It is a novel commercial pinosylvin extract product in development. Retinari™ is obtained from Scots pine wood material through a proprietary raw material treatment and solvent extraction process. The resulting substance subsequently undergoes an affinity chromatography process that enriches the available pine stilbenoids and especially the pinosylvin content in the final product. Retinari™ contains not less than 10% pine stilbenoids (6% weight per weight pinosylvin) among other natural pine phytocompounds. The treatment group was fed with Retinari™, baked into a standard chow, for 10 weeks prior to the ERG recordings while the control group continued with regular chow. Standard chow was ground to homogenous powder and split in half. Geometric dilution was used for adding Retinari™ (1.5% weight per weight) to the other half of chow powder. Water was added for both halves to increase baking quality. Round-shaped balls weighing approximately 13 g were baked from both halves, dried at room temperature, and stored at -20°C. The selected pinosylvin consumption target was set to 50–250 mg/kg/day. The mice were single-housed for the treatment period. Fresh chow with or without Retinari™ was delivered three times a week, and the food consumption was monitored weekly to calculate the pinosylvin intake. The intake was normalised against animal weight.

### 2.2. ERG Recording

Before ERG recordings, the mice were dark-adapted overnight. Preparations for the recordings were performed in the dark with dim red LED-aided flashlights. The mice were anaesthetised using intraperitoneal injections with a mixture of 1.0 mg/kg body weight of medetomidine (Domitor® vet 1 mg/ml, Orion Pharma, Espoo, Finland) and 75 mg/kg body weight of ketamine (Ketalar®/Ketaminol® 50 mg/ml, Pfizer Oy Animal Health, Espoo, Finland) and then placed on a thermal pad in the full-field ERG dome, maintaining body temperature at approximately 38°C. The pupils were dilated with tropicamide (Oftan Tropicamid 5 mg/ml, Santen Pharmaceutical Co., Ltd., Tampere, Finland), and the surface of the cornea was moisturised with carbomer artificial tears (Viscotears 2.0 mg/g, Alcon® a Novartis company). The recordings were conducted first in scotopic, followed by photopic protocol.

The ERG signals were recorded (Espion ERG; Diagnosys LLC, Cambridge, UK) using a gold wire electrode placed on both eyes corneally. The signals were amplified with a band-pass setting of 1–300 Hz for scotopic and 0.3–500 Hz for photopic with a sampling frequency of 2 kHz. A platinum needle reference electrode was placed subcutaneously on the forehead and a platinum needle ground electrode subcutaneously just superiorly from the tailbone. Both eyes were stimulated equally with ColorDome Ganzfeld full-field ERG. The scotopic protocol included recording dark-adapted responses to five distinct stimulus intensities of blue light: 0.003, 0.007, 0.03, 0.5, and 1 Cd × s/m^2^. 15 sweeps of 250 ms at each intensity were recorded with a delay of 10 seconds between each sweep. A 60-second light-adaptation period in 20 Cd/m^2^ white light (6500 K) was applied before the photopic responses. The photopic protocol consisted of light-adapted responses to six distinct stimulus intensities using white light: 0.1, 1, 3, 5, 10, and 20 Cd × s/m^2^ in the presence of continuous background illumination of 20 Cd/m^2^. 25 sweeps of 300 ms were recorded with a delay of 5 seconds between each sweep. An additional 60 seconds of wait time was included between the changes in stimulus intensities. The baseline was set identically for all the recording protocols using the average voltage reading from the duration of 20 ms preceding the stimulus onset. The responses were then exported for off-site analysis.

### 2.3. ERG Signal Processing and Feature Extraction

Postprocessing of the exported ERG data was performed with MATLAB (MathWorks® MATLAB® R2018b). For a-wave analysis, the sweeps were averaged and the a-wave trough was determined as the lowest point of the signal following stimulus onset and preceding the rising phase of the b-wave. The individual sweeps were then low-pass filtered using 5th order Bessel filter with a stopband edge frequency of 60 Hz and then averaged for each stimulus intensity. The b-waves were mapped on the averaged Bessel-filtered signal by fitting a 2nd order polynomial in the surrounding of the highest value of voltage following a-wave. The width of the polynomial was dynamically set as twice the time elapsed from the a-wave trough to the highest voltage point of the signal (initial estimate of b-wave peak). The polynomial fit was iterated five times or until no change in fit parameters occurred, always in the surrounding of the peak of the parabola. All peak fits were visually checked and adjusted manually if determined inaccurate. The b-wave amplitude values were reported as the difference between the determined b-wave peak and a-wave trough. The peak time of each wave was the time elapsed from the stimulus onset until the determined trough (a-wave) or peak (b-wave) of the signal.

### 2.4. OCT Imaging

Following the ERG recordings, OCT was performed on the mice (Phoenix MICRON™ Image-Guided OCT, Phoenix Technology Group, LLC, Pleasanton, CA, USA) to infer total retinal thickness. 50 repetitive images were acquired and averaged. The retinal layers from the averaged OCT images were evaluated by analysis with InSight image segmentation software (Voxeleron LLC, San Francisco, CA, USA). The acquired layer thickness data were then exported for off-site statistical analysis.

### 2.5. Antioxidant Capacity Analysis

The blood samples were collected by cardiac puncture under terminal anaesthesia, which was followed by cervical dislocation and eye enucleation. The blood samples were placed in Eppendorf tubes and stored for coagulation at room temperature for two hours. After coagulation, samples were centrifuged for 15 min (1500 × g) at 4°C and the separated serum was collected for antioxidant capacity analysis.

The Total Antioxidant Capacity Assay Kit (#MAK187, Sigma-Aldrich, St. Louis, MO, USA) was used to measure the total antioxidant capacity as well as small molecule antioxidants by masking the protein activity according to the manufacturer's instructions. Enzymes measured by the kit include catalase (CAT) and peroxidase. The small molecule antioxidants include tocopherols, carotenes, vitamin A, ubiquinols, glutathione, and ascorbate. Briefly, serum samples were diluted with water in a ratio of 1 : 350 to measure total antioxidant capacity. When measuring small molecule antioxidant capacity, the samples were first diluted with Protein Mask solution in a ratio of 1 : 1 and then to a similar concentration as in the total antioxidant capacity measurement. 100 *μ*l of diluted samples were placed on a 96-well plate, and 100 *μ*l of Cu^2+^ Working Solution was added to each well. After the addition of the Cu^2+^ Working Solution, the plate was incubated at room temperature for 90 min. The absorbance of reduced Cu^+^, representing antioxidant capacity by chelation with a colorimetric probe, was recorded using a spectrophotometer (BioTek ELx808, BioTek Instruments, Winooski, VT, USA) at 570 nm. A Trolox standard curve was used for quantitation. The results are presented as Trolox equivalents.

### 2.6. Immunohistochemical Staining

The enucleated eyes were quickly rinsed in PBS (pH 7.4), followed by fixation in 4% paraformaldehyde in 0.1 M phosphate buffer for 24–48 hours and continued with ethanol dehydration and embedded in paraffin. 5 *μ*m thick parasagittal serial sections were cut with a microtome (SM2000 R, Leica, Heidelberg, Germany) for immunohistochemical analysis. The cut tissue sections were deparaffinised using xylene and rehydrated. Then, the glass sections were incubated for 25 min in the dark with 0.5% Sudan Black B (Acros Organics, Morris Plains, NJ, USA) in 70% ethanol. The sections were encircled with a PAP pen and quenched with 0.1 M glycine in PBS for 10 mins prior to a 0.1% Triton-X wash for 10 min before continuing with blocking for 30 min. Quenched slides were incubated with 20% goat serum for 30 min before adding the first primary antibodies (Table 1) and incubated overnight at 4°C. The sections were incubated at room temperature for 30 min and washed in the dark for 10 min. Then, the first secondary antibodies were added and incubated for 3 hr. Finally, DAPI (Sigma-Aldrich, St. Louis, MO, USA) was added at a ratio of 1 : 10 000 and incubated for 30 min followed by 5 min wash with TBS. Then, the slides were mounted using Mowiol mounting media and stored in the dark at room temperature. The correct location near the optic nerve and the quality of the sections were monitored with haematoxylin and eosin (H&E) staining.

The secondary antibodies were Goat anti-Rabbit Alexa Fluor 594 (A11037) and Goat anti-Mouse Alexa Fluor 594 (A11032) (ThermoFisher Scientific, Waltham, MA, USA) diluted at 1 : 500.

### 2.7. Confocal Imaging

The RPE layer of the stained sections was examined with a confocal microscope (Zeiss AX10 Imager A2, Zeiss, Germany) using a 63x (NA:1.42. Plan Apochromat) oil (Zeiss Immersol™, Germany) immersion objective. The microscopy settings were kept identical for all pictures taken and held constant during imaging. Representative high-power microphotos were taken close to the vicinity of the optic nerve with ZEN blue v2.3 (Carl Zeiss Microscopy, Germany). At least nine repetitive images were taken per animal, and several regions of interest were analysed per view and averaged. All the captured images were processed using ImageJ (version 1.52a). The background was subtracted using a default rolling ball radius method. Regions of interest (ROIs) were drawn followed by mean grey-value measurement. ROIs were kept constant within each antibody analysed. All the imaging analyses were blindly quantified at least by 3 independent researchers. The number of biological replicates per group varied between four and five (Table 2). Images were color enhanced using Adobe Photoshop® for visual representation.

### 2.8. Statistics

The statistical analysis and plotting of the ERG results were done with R (version 3.5.3). The regular two-way analysis of variance (ANOVA) was used to infer statistical significance for each stimulus intensity with Bonferroni correction. The main effect between each treatment group and the genotype was determined by two-way ANOVA using the genotype and stimulus intensity as independent variables. If significance was determined, the test was followed by the Bonferroni *post hoc* test with multiple pair-wise comparisons using Student's *t*-test. The statistical analysis for the OCT and serum antioxidant capacity data was also determined with Student's *t*-test. The Mann–Whitney *U* test was used in the immunohistochemical staining analysis. Values of *p* < 0.05 were considered significant. Data are presented as the mean ± standard deviation (SD). Both eyes were utilised in the statistical analysis of ERG, OCT, and immunohistochemical staining.

## 3. Results

### 3.1. Retinari™ Consumption

The subpopulation size, age distribution, and pinosylvin intake for each group are reported in Table 2. The average pinosylvin consumption in all treated mice was 141.5 ± 17.0 mg/kg/day. The WT mice consumed 138.7 ± 19.0 mg/kg/day of pinosylvin, and the NFE2L2 KO mice consumed 147.1 ± 9.8 mg/kg/day for the 10 weeks. No statistical differences were observed between the ages of each study group nor in the pinosylvin consumption between the WT and NFE2L2 KO mice.

### 3.2. Retinari™ Preserves Retinal Function of the NFE2L2 KO Mice in Scotopic ERG

The scotopic a- and b-wave amplitudes of the NFE2L2 KO control mice were substantially smaller than those of the WT treated and control groups (dashed red and black lines in Figures 1(a)–1(d); *p* < 0.001 for each group), suggesting accelerated retinal degeneration in the NFE2L2 KO mice compared to the WT mice. However, the 10-week-long Retinari™ treatment more than doubled both the scotopic a- and b-wave amplitudes in the NFE2L2 KO mice while it had only a minor effect on the a- and b-wave amplitudes of the WT mice. The relative increase in the a- and b-wave amplitudes in the NFE2L2 KO treated mice was highly significant (Figures 1(a) and 1(b); *p* < 0.001 for both waves), surpassing the amplitudes of even the WT control group. This would seem to suggest that Retinari™ prevents the negative degenerative changes in the NFE2L2 KO mice from occurring.

### 3.3. Retinari™ Preserves Retinal Function of the NFE2L2 KO Mice in Photopic ERG

Similarly, as in the scotopic ERG, also the photopic ERG demonstrated more inferior b-wave amplitudes in the NFE2L2 KO control group than the WT control group, although this was not statistically significant (Figure 2). While the photopic WT mouse b-wave amplitudes were preserved at the same level in treatment and control groups, the NFE2L2 KO treated mice surpassed the values of WT treated (*p* < 0.05), WT control (*p* < 0.01), and NFE2L2 KO control (*p* < 0.001) mice. This indicates diminished levels of degeneration in retinal function.

### 3.4. Retinari™ Preserves the Retinal Thickness in NFE2L2 KO Mice

Ten-week-long Retinari™ treatment of NFE2L2 KO mice resulted in significantly higher total retinal thickness (TRT; Figure 3) as measured from the retinal nerve fibre layer (RNFL) to RPE (*p* < 0.01). TRT in the WT control group was significantly thicker than in the NFE2L2 KO control group (*p* < 0.05). The WT treated mice had visibly increased TRT compared to the WT control group, although this did not reach a statistical significance.

### 3.5. Retinari™ Treatment Enhances Serum Antioxidant Enzyme Capacity in WT Mice

After attaining clear electrophysiological and morphological results in favour of the Retinari™ treatment, we wished to analyse its systemic effect on antioxidative mechanisms. The WT mouse serum samples showed increased enzyme-derived antioxidant capacity after 10 weeks of Retinari™ treatment (Figure 4(a); *p* < 0.01). Simultaneously, the capacity of small molecule antioxidants reduced (*p* < 0.05) resulting in no change in total antioxidant capacity. NFE2L2 KO mice showed no response to the Retinari™ treatment. Instead, the antioxidant capacities of small molecule antioxidants and protein antioxidants remained at a basal level (Figure 4(b)).

### 3.6. Long-Term Retinari™ Treatment Increased Antioxidant Levels in the RPE Layer in NFE2L2 KO Mice

Since the serum data on the antioxidant capacity revealed no systemic benefits for the NFE2L2 KO mice in contrast to our ERG and OCT findings, we proceeded to analyse the levels of antioxidants directly in the RPE layer. As a result of the 10-week-long Retinari™ treatment, highly significant increases in the levels of the antioxidant enzymes superoxide dismutase 1 (SOD1) and CAT were detected in NFE2L2 KO mice (Figure 5; *p* < 0.001 for both). The increased levels of SOD1 and CAT implicate upregulated antioxidant capacity in the RPE. WT mice also exhibited increased values for SOD1 (*p* < 0.001) and CAT (*p* < 0.01).

### 3.7. Long-Term Retinari™ Treatment Increased p62, Ubiquitin, and LC3B Levels in the RPE Layer of WT Mice but Decreased Ubiquitin Content in the RPE Layer of NFE2L2 KO Mice

After 10 weeks of Retinari™ treatment, immunohistochemical analysis of the RPE layer of WT mice revealed an increase in ubiquitin (*p* < 0.001) and p62 (*p* < 0.001), markers of proteins destined for degradation and protein aggregates, respectively (Figures 6(a) and 6(b)). However, the mice showed an increase in autophagosome marker LC3 (*p* < 0.001) as well, suggesting a decrease in autophagic degradation. The marker of lipid oxidation, 4-HNE, showed no change between the control and Retinari™ treated WT mice. The decrease of autophagy activity after Retinari™ treatment did not evoke oxidative stress. The NFE2L2 KO mice showed a decreased level of ubiquitin (*p* < 0.05) after Retinari™ treatment (Figures 6(c) and 6(d)). However, the autophagy markers p62 and LC3 and lipid oxidation marker 4-HNE remained at a basal level.

### 3.8. Long-Term Retinari™ Treatment Decreased Inflammation in the RPE Layer in NFE2L2 KO Mice

The inflammation marker, CRP, levels increased in the retina of WT mice (Figures 7(a) and 7(b); *p* < 0.01) and had an even higher increase in the RPE layer (Figure 7(c); *p* < 0.001). In contrast, CFH levels experienced a highly significant decrease in the retina of WT mice as a response to the treatment (Figures 7(b); *p* < 0.001), whereas the change was nonsignificant when observed in the RPE layer (Figure 7(c)). For the NFE2L2 KO mice, CRP levels remained unchanged in treated mice in the retina and RPE layer (Figures 7(d)–7(f)). A highly significant increase in CFH levels was detected in the retina in response to the treatment (Figure 7(e); *p* < 0.001). When examined in the RPE layer, a similar relative increase was detected (Figure 7(f); *p* < 0.05). Since CRP and CFH are related to each other in an inverse relationship in AMD retinas, the results seem to suggest that the retina of the WT mice experienced slightly increased inflammation in treated individuals. On the other hand, the clear CFH increase in the retina and RPE layer of NFE2L2 KO mice treated individuals suggests a possible protective effect against chronic inflammation, although the change was not observed in the CRP levels.

## 4. Discussion

In this study, pinosylvin was administered as a standardised natural extract from pinewood material, named Retinari™. Specifically of interest were the effects of Retinari™ on the NFE2L2 KO mice, a phenotype with dry AMD-like changes in the retina. Previous studies have introduced pinosylvin via intraperitoneal injections ranging from 10 to 100 mg/kg as a single dose [42] and 2–10 mg/kg/day in a 10-day-long experiment [37, 43]. Studies with the enteral introduction of resveratrol on mice have shown beneficial effects at concentrations of 50–250 mg/kg/day [44–46]. Furthermore, one study investigated 50 mg/kg/day oral pinosylvin, finding systemic effect on antioxidant defence after 28 days of treatment [47]. However, because the transfer of the observed molecular changes onto the retinal function might take longer, we set our treatment duration to 10 weeks. Subsequently, our target consumption of pinosylvin was 50–250 mg/kg/day.

There was a significant baseline difference in ERG and TRT between WT and NFE2L2 KO control mice with the latter showing lowered a- and b-wave amplitudes in scotopic ERG and thinner retina. A similar baseline difference was observed for photopic ERG b-wave amplitude values. The a-wave stems mainly from the photoreceptor cells, and its reduction has been connected to AMD, especially in the late stages [48–50]. Thus, the reduced retinal function and decreased TRT are indicative of higher retinal dysfunction in NFE2L2 KO mice. This is in line with previous knowledge of the detrimental effects of the lack of the *NFE2L2* gene on retinal function [41]. NFE2L2 KO mice, despite their lower baseline retinal function and thinner TRT compared to WT, responded remarkably well to Retinari™ treatment. The Retinari™ treated NFE2L2 KO mice presented with a highly significant increase of scotopic a- and b-wave amplitudes as well as thicker TRT in OCT. A similar increase was observed for photopic ERG b-wave amplitudes. Previous studies reveal that resveratrol increases b-wave amplitudes and contributes to a thicker outer nuclear layer in the aged mouse retina [51, 52]. Retinal thickness across the retina has been shown to decrease with age [53], and it is related to AMD progression [54, 55]. Our results suggest a strong protective effect of Retinari™ against the gradual decline of retinal function observed in ageing and the dry AMD mouse models.

Due to significantly improved retinal function discovered in NFE2L2 KO mice and directional improvements in WT mice, we studied the possible molecular factors involved in these changes first by measuring antioxidant levels from the serum. The treatment in WT mice yielded higher protein antioxidant capacity. However, there was no change in the total antioxidant capacity. We have previously demonstrated pinosylvin to function as an antioxidant defence system enhancer in human RPE cells (ARPE-19) via activating NFE2L2, a master regulator of antioxidant defence [38]. Several antioxidant enzymes are under the control of NFE2L2 [12–14]; therefore, the increase in the serum antioxidant enzyme capacity supports the results gained from *in vitro* work. However, the antioxidant defence system is strictly regulated to sustain redox homeostasis, a balanced environment for normal biological functions [56]. The increased antioxidant defence may lead to reductive stress, and therefore, the system would need to be balanced. In this case, the treated mice seemed to reduce small molecular antioxidants in their serum to balance the redox environment. Despite the similar outcomes in total antioxidant capacity between the controls and the treated mice, antioxidant enzymes can be considered more efficient in combating oxidative stress. This is due to their ability to neutralise free radicals at the site of origin and function repetitively, whereas nonenzymatic antioxidants mainly protect from ongoing free radical chain reactions [57]. The desirable systemic effect seen in WT mice was not observable in NFE2L2 KO mice. Due to the clear ERG findings in preserving the retinal function of NFE2L2 KO treated mice, we anticipated local Retinari™ effects on the retina. This led us to inspect RPE-level effects where we found a clear increase in the expression of antioxidant enzymes SOD1 and CAT in the RPE layer of the treated NFE2L2 KO mice. Increases were also detected for the WT mice, although CAT levels experienced a slightly lower relative increase than the NFE2L2 KO mice. Since the NFE2L2 KO mice lack NFE2L2, the primary target of pinosylvin, but still demonstrate an enhancement of antioxidant defence, the potential antioxidant defence upregulation effect may arise from one of the metabolites of pinosylvin: resveratrol [35, 36]. Resveratrol exhibits neuroprotection through increased superoxide dismutase 2 and thioredoxin 2 production when exposed to a neurotoxin [58, 59]. Furthermore, SOD1 upregulation is not generally considered a result of NFE2L2 activation whereas CAT seems to be directly controlled by NFE2L2 [17]. Known targets of resveratrol, AP-1, and FoxO on the other hand can induce both SOD1 and CAT expression [17, 39, 40]. In addition, although pinosylvin has been found to act via NFE2L2 signalling *in vitro* [38], other possible targets cannot be ruled out, especially for *in vivo* models. Therefore, it seems convincing that Retinari™ upregulates local antioxidant enzyme production in the RPE which is the primary site affected in AMD pathogenesis and the site experiencing high rates of oxidative stress in the retina.

In addition to upregulated antioxidant enzyme levels, a possible mechanism of Retinari™ is elicited via the autophagy clearance system. The increase of ubiquitin and p62 in the RPE layer of the treated WT mice suggests reduced autophagic activity as well as accumulation of ubiquitin-conjugated proteins and protein aggregates. However, increased LC3 levels imply still functional autophagy due to the formation of autophagosomes, suggesting rather downregulation of autophagic degradation than inhibition. In contrast, Retinari™ treatment of NFE2L2 KO mice showed a decrease in ubiquitin content in RPE cells. However, the markers of autophagy activity remained at a basal level. Autophagy can be considered a part of the antioxidant defence system [60–62], and therefore, its downregulation may serve as a marker of increased antioxidant defence. In fact, long-term NFE2L2 activation has been shown to decrease autophagy [63], and the role of NFE2L2 on the regulation of autophagy shows dynamic adaptation to environmental conditions [64]. On the other hand, if the antioxidant defence system is enhanced by Retinari™, there might not be material for autophagic degradation due to reduced oxidative stress. Recently, pinosylvin has been found to protect from cerebral ischemia by activating antioxidant defence via NFE2L2 and mitophagy, a selective form of autophagy to remove dysfunctional mitochondria, resulting in decreased oxidative stress due to enhanced antioxidant defence and removal of reactive oxygen species- (ROS-) leaking mitochondria [65].

The inflammatory marker CRP was not affected in NFE2L2 KO mice as a result of the treatment but was interestingly increased in the WT mouse RPE cells and the entire retina. The CRP increase in WT mice could be explained by a host defence stress reaction to polyphenolic Retinari™. Since NFE2L2 KO shows upregulated stress markers, CRP elevation is not needed anymore or its production is suppressed [8]. The CFH levels, on the other hand, climbed in the RPE cells and the retina as a whole in the NFE2L2 KO mice. It is well known that CFH inhibits the alternative complement pathway [23]. Our observations reveal that Retinari™ reduces complement system-mediated tissue inflammation in the retina including the RPE cells of NFE2L2 KO mice. The WT mice were found to have reduced retinal CFH levels while remaining at basal levels in the RPE cells. Polyphenolic compounds, including resveratrol, inflict low-level stress reaction within normal cells [66]. Such stress is beneficial in combating oxidative stress and enhancing autophagic clearance. Taken together, the apparent inflammatory marker increase is not alarming, considering that the absolute levels are very low in the untreated WT mice. The stress levels of NFE2L2 KO mice, on the other hand, are already at such a high state initially that the effect seems to be rather a reduction in inflammation.

Since Retinari™ contains approximately 6% pinosylvin, it cannot be conclusively determined whether pinosylvin alone or its metabolite, resveratrol, as a cocontributor, explains our findings. More importantly, it is clear that Retinari™ elicits a positive impact on the NFE2L2 KO mice. Although it contains a large proportion of other phytochemicals and wood-derived material, pinosylvin and resveratrol are the most likely compounds explaining our findings due to their known role in antioxidative defence and autophagy. For example, pinosylvin is able to reduce nitrosative stress and enhance removal of ROS generating damaged mitochondria having an impact on total oxidative stress met in the cell [65, 67]. Resveratrol in turn has been linked to antioxidant defence and autophagy enhancement as well as inflammatory response regulation, including CFH-linked complement system modulation [40, 68, 69]. Furthermore, improved ERG function has also been associated with resveratrol in aged rats [70] and mice with light-induced retinal degeneration [51, 52]. All molecular characteristics mentioned above are in logical continuum generating a treadmill worsening the situation on the retina in every turn. Increased oxidative stress creates a demand for efficient removal of damaged proteins and cell organelles. When damaged material starts to accumulate creating more oxidative stress due to insufficient removal, cellular wellbeing is compromised leading to cell death and inflammatory response [71]. These molecular changes can be traced to AMD at a local and systemic level [72]. Increased oxidative stress can be seen as the trigger of this damaging cycle; therefore, oxidative stress limiting strategies, not forgetting treatment of its aggravating factors, including dysfunctional autophagy and inflammation, are of interest.

## 5. Conclusions

Our study demonstrates the positive impact of Retinari™ treatment as an effective polyphenolic extract on the retinal function and TRT of NFE2L2 KO mice. This effect is likely mediated by local effects in the RPE layer, such as enhanced antioxidant enzyme activity by CAT and SOD1 as well as by reduced chronic inflammation as indicated by the increased CFH levels. The main benefits of pinosylvin-containing Retinari™ include its vast availability in nature in comparison to pinosylvin's thought analogue, resveratrol, its consecutive affordability in concern to extraction and production to dietary supplement, and its metabolism to resveratrol *in vivo*. We hypothesise that patients with increased risk factors for developing AMD could benefit from oral Retinari™ supplementation to slow down the degenerative disease onset by inflicting its main positive effects on antioxidant enzyme production and locally reduced chronic inflammation. Even patients with AMD could potentially benefit from the supplement by improving retinal function and defence against age-related oxidative stress. Clinical trials for Retinari™ for AMD are highly anticipated.

## Figures and Tables

**Figure 1:** Scotopic ERG in the Retinari™ treatment trial. The treated mice were fed Retinari™ for 10 weeks prior to ERG while controls received regular chow. (a) The ERG a-wave amplitudes of NFE2L2 KO Retinari™ treated mice (*n* = 5) increased significantly compared to the control mice (*n* = 5). WT mice had no significant effects between the treatment group (*n* = 4) and the control group (*n* = 5). (b) b-wave amplitudes were significantly higher in NFE2L2 KO Retinari™ treated mice versus NFE2L2 KO and WT control mice. The NFE2L2 KO control group had significantly lower amplitudes than the other genotypes' controls and WT treatment group. (c) Averaged raw ERG signals of each group at a flash intensity of 0.03 Cd × s/m^2^. (d) Filtered (5th order low-pass Bessel filter with a cut-off at 60 Hz) ERG signals of the same responses as in (c). The b-wave location was determined from the filtered signal. ^∗^*p* < 0.05, ^∗∗^*p* < 0.01, and^∗∗∗^*p* < 0.001, Student's *t*-test.

**Figure 2:** Photopic ERG in the Retinari™ treatment trial. The treated mice were fed Retinari™ for 10 weeks prior to ERG while controls received regular chow. (a) The ERG b-wave amplitudes of WT Retinari™ treated mice (*n* = 4) experienced no significant differences compared to the control mice (*n* = 5). b-wave amplitudes were significantly higher in NFE2L2 KO Retinari™ treated mice (*n* = 5) compared to the NFE2L2 KO control (*n* = 5), WT control, and WT treated groups. (b) Averaged raw ERG signals of each group at a flash intensity of 5 Cd × s/m^2^. (c) Filtered (5th order low-pass Bessel filter with a cut-off at 60 Hz) ERG signals of the same responses as in (b). ^∗^*p* < 0.05 and^∗∗^*p* < 0.01, Student's *t*-test.

**Figure 3:** OCT in Retinari™ treatment trial. (a) Representation of the total retinal thickness as measured from the RNFL to RPE. A significant increase was inferred for NFE2L2 KO treated (*n* = 5) with Retinari™ in comparison to the control group (*n* = 5). The WT control group (*n* = 5) had a significantly higher total retinal thickness than the NFE2L2 KO control group (*n* = 4). (b) Representative OCT images of control and treated WT and NFE2L2 KO mice. The scale bar indicates 100 *μ*m. (c) Representative microscope images (20x) of H&E-stained mouse retinas from control and treated WT and NFE2L2 KO mice. GCL = ganglion cell layer; INL = inner nuclear layer; IPL = inner plexiform layer; ONL = outer nuclear layer; OPL = outer plexiform layer; PL = photoreceptor layer; RPE = retinal pigment epithelium. The scale bar indicates 20 *μ*m. ^∗^*p* < 0.05 and ^∗∗^*p* < 0.01, Student's *t*-test.

**Figure 4:** Serum antioxidant assay. Retinari™ increased serum protein antioxidant capacity of WT treated mice (*n* = 4) compared to the WT control mice (*n* = 5) without affecting total antioxidant capacity. No differences were detected in NFE2L2 treated (*n* = 5) individuals in comparison to the control mice (*n* = 5). Serum total antioxidant, small molecular antioxidant, and protein antioxidant capacities of (a) WT mice and (b) NFE2L2 KO mice expressed in mM Trolox equivalent after 10 weeks of Retinari™ treatment. ^∗^*p* < 0.05, Student's *t*-test.

**Figure 5:** Immunohistochemical staining of antioxidant activity in the RPE cells. (a) Representative high-power confocal microscopy images of SOD1 and CAT in a WT mouse. (b) The treated WT mice (*n* = 4) exhibited increased levels of SOD1 and CAT in the RPE layer when compared to the control mice (*n* = 5). (c) Representative high-power confocal microscopy images of SOD1 and CAT in an NFE2L2 KO mouse. (d) The SOD1 and CAT levels were enhanced in treated individuals (*n* = 5) than in control (*n* = 5) NFE2L2 KO mice. Scale = 5 *μ*m. ^∗∗^*p* < 0.01 and^∗∗∗^*p* < 0.001, Mann–Whitney *U* test.

**Figure 6:** Immunohistochemical staining of autophagy markers in the RPE cells. (a) Representative high-power confocal microscopy images of p62, LC3B, ubiquitin, and 4-HNE in a WT mouse. (b) The treated (*n* = 4) WT mice exhibited increased levels of p62, LC3B, and ubiquitin in the retina compared to the control mice (*n* = 5). The 4-HNE levels slightly decreased in response to treatment. (c) Representative high-power confocal microscopy images of p62, LC3B, ubiquitin, and 4-HNE in an NFE2L2 KO mouse. (d) The ubiquitin levels were higher in NFE2L2 KO control (*n* = 5) than in treated (*n* = 5) mice. The levels of p62 and LC3B showed a marginal increase and 4-HNE a marginal decrease in treatment groups. Scale = 5 *μ*m. ^∗^*p* < 0.05 and ^∗∗∗^*p* < 0.001, Mann–Whitney *U* test.

**Figure 7:** Immunohistochemical staining of inflammation markers across the whole retina and in the RPE cells. (a) Representative high-power retinal cross-section microscopy images of CRP and CFH in a WT mouse retina. (b) The treated (*n* = 4) WT mice exhibited increased retinal levels of CRP and decreased CFH levels compared to the control mice (*n* = 5). (c) In the RPE layer, CRP was similarly increased in WT mice, but CFH remained at basal levels. (d) Representative high-power retinal cross-section microscopy images of CRP and CFH in an NFE2L2 KO mouse. (e) The retinal levels of CRP were unaffected, and the CFH levels were enhanced in treated (*n* = 5) NFE2L2 KO individuals in comparison to controls (*n* = 5). (f) In the RPE layer, CRP remained at basal levels in NFE2L2 KO mice while CFH was slightly higher in treated individuals. Scale = 10 *μ*m. GCL = ganglion cell layer; INL = inner nuclear layer; ONL = outer nuclear layer. ^∗^*p* < 0.05,  ^∗∗^*p* < 0.01, and^∗∗∗^*p* < 0.001, Mann–Whitney *U* test.

**Table 1:** List of primary antibodies.

Primary antibodies against	Isotope	Working dilution	Supplier/catalogue number
p62	Polyclonal	1 : 100	CT-5114
LC3B	Monoclonal	1 : 100	CT-3868
Ubiquitin	Monoclonal	1 : 100	CT-3936
4-HNE	Polyclonal	1 : 100	LS-C68182
SOD1	Polyclonal	1 : 100	ab13498
CAT	Polyclonal	1 : 100	ab16731
CRP	Polyclonal	1 : 100	ab65842
CFH	Monoclonal	1 : 50	NBP2-90802

**Table 2:** The genotype- and trial group-specific sample sizes, age distribution, and pinosylvin intake.

Genotype	Trial group	*n*	Age	Pinosylvin intake
WT	Control	5	16.5 ± 3.6 months	0 mg/kg/day
	Treatment	4	15.2 ± 2.6 months	138.7 ± 19.0 mg/kg/day

NFE2L2 KO	Control	5	15.2 ± 4.0 months	0 mg/kg/day
	Treatment	5	15.3 ± 4.5 months	147.1 ± 9.8 mg/kg/day

## Data Availability

The data presented in this study are available on request from the corresponding author.

## Supplementary Materials

Supplementary Materials Figure S1: weekly chow consumption. Figure S2: original 63x oil immersion images of the autophagy marker staining. Figure S3: original 63x oil immersion images of the antioxidant activity staining. Figure S4: original haematoxylin and eosin stains of the retina.
